# Cognition/Psychological Burden and Resilience in Cutaneous T-Cell Lymphoma and Psoriasis Patients: Real-Life Data and Implications for the Treatment

**DOI:** 10.1155/2022/8802469

**Published:** 2022-07-21

**Authors:** Giovanni Damiani, Joselin D. Tacastacas, Timothy Wuerz, Lindsay Miller, Philip Fastenau, Christopher Bailey, Mansi Sethi Chawa, Amanda Argenas, Marco Fiore, Kevin D. Cooper, Alan J. Lerner

**Affiliations:** ^1^Department of Dermatology, University Hospitals Cleveland Medical Center, And Case Western Reserve University, Cleveland, OH, USA; ^2^Department of Biomedical, Surgical and Dental Sciences, University of Milan, Milan, Italy; ^3^Department of Psychiatry, Henry Ford Hospitals, Detroit, MI, USA; ^4^Department of Neurology, University Hospitals Cleveland Medical Center, Cleveland, OH, USA; ^5^Los Angeles County Department of Mental Health, Redondo Beach, CA, USA; ^6^Department of Dermatology, University Hospitals Cleveland Medical Center, Cleveland, OH, USA; ^7^Department of Critical Care Medicine, University of Pittsburgh School of Medicine, Pittsburgh, PA, USA; ^8^Department of Women, Child and General and Specialized Surgery, University of Campania “Luigi Vanvitelli”, Naples, Italy

## Abstract

**Background:**

Psoriasis and cutaneous T-cell lymphoma (CTCL) expose patients to chronic inflammation as well as physical and psychological disabilities, but the impact of such alterations on cognitive function is unknown.

**Objective:**

This study is aimed at determining if CTCL and psoriasis impact cognitive functioning in relation to psychological and health-related quality of life (HR-QOL) status.

**Methods:**

A cross-sectional study was performed in an outpatient dermatology clinic of a university teaching hospital. Thirty-nine subjects with CTCL (*N* = 20) or psoriasis (*N* = 19) who met eligibility criteria were included. The cognitive domains of memory, attention and processing speed, and executive function were assessed with standard neuropsychological tests. Subjects were assessed for depression, anxiety, and HR-QOL (using the SKINDEX-29 questionnaire).

**Results:**

Study participants were CTCL and psoriasis subjects; cognitive impairment was found in the domain of memory in 17.9% subjects with CTCL or psoriasis. Lower scores on executive function tests were predicted by higher (worse HR-QOL) SKINDEX-29 functioning scores (*p* = 0.01). A higher estimated baseline intellectual functioning predicted lower scores (better HR-QOL) on the symptoms and functioning domains of SKINDEX-29 (*p* = 0.01 and 0.02, respectively) and a statistical trend (*p* = 0.07) for the emotion domain. Memory and acute anxiety were adversely impacted by shorter disease duration (*p* = 0.01 for both).

**Conclusions:**

Memory impairment may be associated comorbidity in CTCL and psoriasis. Subjects with stronger cognitive resources appear to cope better with health-related quality of life (HR-QOL) challenges.

## 1. Introduction

Chronic skin diseases, both inflammatory and neoplastic, may couple with a systemic inflammatory status leading to physical and psychological disabilities [1–3]. The real impact of systemic inflammation on cognitive function is still debated, and few dermatological studies have explored this link; however, differences in both methods and subsets of analyzed patients make their comparison problematic [4–8]. Interestingly, both skin diseases and mild cognitive impairment (MCI) contribute to decreased HR-QOL [9], defined as a person's subjective assessment of the ability to function and pursue valued life goals in several domains including physical functioning, somatic sensations (e.g., pain or pruritus), psychological (e.g., depression and anxiety) and social functioning, and engagement in productive activities, in several different manners [10].

Recent studies shed light on the mechanisms that may trigger early mild cognitive impairment, suggesting a prominent role of T-cells and in particular Th-17 [11] and also of neutrophil adhesion in brain capillaries provoking a blood flow reduction [12]. Concordantly, T-cells play a pivotal role in the pathogenesis of psoriasis [11] and in the progression of cutaneous T-cell lymphoma (CTCL) [13]. In addition, physiologic parameters associated with cognitive function such as beta-amyloid accumulation in a transgenic mouse model of Alzheimer's disease were reported to be prevented/reversed by systemic retinoids, which are used in both psoriasis and CTCL [14]. Both CTCL and psoriasis patients often present with cardiovascular and metabolic comorbidities, which also are capable of increasing the risk of early cognitive impairment and MCI [15].

The aim of the present study was to evaluate, in a selected cohort of CTCL and psoriasis patients, cognitive functioning in relation to physical skin disease burden, psychological status, and HR-QOL status.

## 2. Methods

### 2.1. Study Population

In this cross-sectional study, subjects were randomly recruited from the outpatient dermatology clinics of a university teaching hospital following University Hospitals Cleveland Medical Center institutional review board approval. The randomization was performed with a random number table.

In accordance with Petersen criteria, we defined mild cognitive impairment (memory, attention/processing speed, and executive function) as a low performance > 1.5 SD below the mean in one or more cognitive domains adjusted for age and educational background not otherwise explained with delirium or other psychiatric disorders that do not substantially interfere with daily activities [15].

Inclusion criteria included age of at least 40 years (Since the majority of CTCL cases are diagnosed between 40 and 60 y, we decided to set this temporal inclusion criterion also for psoriatic patients to increase the comparability.), fluency in English, at least 8 years of formal education, biopsy-confirmed CTCL, and duration for more than 6 months or clinical diagnosis of psoriasis for more than 6 months.

Exclusion criteria were current or past history within two years of psychiatric diagnosis that meet the Diagnostic and Statistical Manual of Mental Disorders- (DSM-) V criteria for major axis II disorders including psychosis, major depression, bipolar disorder, or neurologic disorder (epilepsy, seizure, focal brain lesion, head injury with loss of consciousness, clinically significant stroke, etc.) that could influence cognitive functioning, history of alcohol or substance abuse or history of rapidly progressive dementia, sensory impairment which would prevent the subject from participating in the study, and history of lymphoma with central nervous system involvement.

### 2.2. Subject Evaluations

Medical and pharmacological history was obtained followed by neuropsychological assessments. The severity of disease for CTCL and psoriasis subjects was measured with the modified Severity-Weighted Assessment Tool (SWAT) [16] and Psoriasis Area and Severity Index (PASI) [17].

### 2.3. Cognitive Parameters

Subjects underwent a battery of well-established standard neuropsychological measures. In order to avoid a potential adaptive mechanism, tests were performed for the first time on every patient with a new physician not previously met in a nonfamiliar room to the patients.

#### 2.3.1. North American Adult Reading Test (NAART)

NAART is used to estimate the level of functioning prior to the onset of a neurological disorder (estimated premorbid intellectual functioning or intelligence quotient). The average mean intelligence quotient is 100 ± 15 points. Performance correlates highly with verbal intellectual ability and is preserved even following significant neurocognitive decline [18, 19].

#### 2.3.2. Memory

Memory was assessed by the Rey Auditory Verbal Learning Test (RAVLT) [20]. The examiner reads a 15-item word list at a fixed rate and requires the examinees to repeat as many words as they can remember after each of 5 presentations; the sum of the 5 trials provides a sensitive index of efficiency of acquisition. Recall is tested again after the examinee is required to repeat a distraction list (List B) and again 30 minutes later (Delayed Free Recall), followed immediately by a Recognition Trial (discriminating the original 15 targets from 35 distractors).

#### 2.3.3. Attention and Processing Speed

This was evaluated by the Stroop Color and Word Test, Trail Making Test parts A and B, and the Wechsler Adult Intelligence Scale-IV (WAIS-IV) Digit Span and Coding subtests. In particular, WAIS-IV scores classified patients into 7 clusters: “very superior” with >129 points, “superior” with 120-129 points, “high average” with 110-119 points, “average” with 90-109 points, “low average” with 80-89 points, “borderline” with 70-79 points, and “extremely low” below 70 points. The Stroop Color and Word Test is a quick screening of rapid automatic naming and mental processing speed (Word and Color Trials) and of response inhibition, an executive skill (Color-Word Trial and Interference Index) [21]. The Trail Making Test parts A and B measures visual scanning, processing speed, and executive functioning with mental flexibility [21]. The WAIS Digit Span measures concentration and very brief memory span by presenting a series of single-digit numbers and having the examinee repeat them back in the same order or in reverse order. The WAIS Digit Symbol measures visual scanning, mental processing speed, and integration of visual input with fine motor execution [21].

#### 2.3.4. Executive Function

This was assessed with the Controlled Oral Word Association Test (COWAT, also known as FAS), Trail Making Test part B, and the Interference Index portion of the Stroop Color and Word Test. The COWAT measures the speed with which an individual can rapidly generate words that fit a particular criterion. Both components (phonemic/letter fluency and semantic/category fluency) measure processing speed, but semantic fluency also measures semantic processing [22].

The animal naming test measures language and frontal/executive functions. The subject is asked to produce as many animal names as possible within 60 seconds [21]. This was the only language test performed.

### 2.4. Psychological Parameters and Health-Related Quality of Life Measures

Measures of depression and anxiety were the Beck Depression Inventory-II (BDI-II) [23] and the State-Trait Anxiety Inventory (STAI), respectively [24]. Higher BDI-II, STAI-state, and STAI-trait scores indicate worse depression, acute anxiety, and chronic anxiety, respectively. In particular, BDI-II values 0-9 are within normal limits, converse values greater than 9 indicate depression (10-15: minimal depression, 16-19: mild to moderate depression, 20-29: moderate to severe depression, and 30+: severe depression). STAI scores range from 20 to 80 points, classifying individuals with 20-37 as affected by “no or low anxiety,” with 38-44 as with “moderate anxiety” and with a score greater than 44 as affected by “high anxiety.”

The SKINDEX-29 is a reliable and valid 29-item questionnaire to measure and evaluate the health-related quality of life (HR-QOL) of patients with skin diseases [25]. In clinical practice, physicians adopted a score ≥ 52 points on symptoms, ≥39 on emotions, ≥37 on functioning, and ≥44 on the overall score to identify a very severe impact on HR-QOL. Results are reported as 3-scale scores assessing 3 domains, namely, emotions, physical symptoms, and functioning, with higher scores indicating worse HR-QOL. Meaningful interpretation is done by comparison of current study scores with previously reported values for other skin diseases, instead of classifying patients into severity categories based on disparate cut-off scores (anchor-based and distribution-based methods) [25–27].

The study fulfilled the principles of the Helsinki declaration and was approved by our institutional review board.

### 2.5. Statistical Analysis

Raw neuropsychological assessment scores were corrected for age and, when possible, gender and education using well-established normative data that are consistent with standard clinical practice in neuropsychology. Composite scores were then created by averaging all the scores within each cognitive domain (memory, attention/processing speed, and executive function). The frequency of cognitive impairment was determined by calculating the percentage of individuals whose cognitive domain scores were greater than 1.5 standard deviations below the normative mean scores, as is consistent in clinical practice. The independent-sample *t*-test and chi-squared/Fisher's exact test were used to examine group differences in demographic and clinical characteristics. ANOVA was used to examine differences in neuropsychological test performance between groups; the exception was the MMSE for which ANCOVA (controlling for age) was used. Linear regression was used to identify potential predictors of cognitive function domains (memory, attention/processing speed, and executive function), SKINDEX-29 domain scores (emotions, symptoms, and functioning), and psychological function (depression, state anxiety, and trait anxiety). Statistical analysis was performed using the IBM Statistical Package for the Social Sciences 23 software.

## 3. Results

### 3.1. Demographics

Forty-two subjects were recruited. One subject with psoriasis was excluded from data analysis because of an invalid neuropsychological assessment due to chronic use of benzodiazepines. Two other subjects with coexisting CTCL and psoriasis confirmed by biopsies were also excluded. Characteristics of the 39 remaining subjects are shown in Table 1 and Figure 1. CTCL subjects were significantly older than psoriasis subjects. There were more married CTCL than psoriasis subjects. Psoriasis subjects had significantly longer mean disease duration compared to CTCL. The mean diastolic blood pressure of psoriasis subjects was significantly higher than CTCL. Seven of 20 subjects with CTCL had prior oral bexarotene therapy.

### 3.2. Cognitive Profile

There were no group differences in cognitive functioning between psoriasis and CTCL subjects (see Table 2 and Figure 2). When the groups were combined for further analyses, cognitive impairment was found in the domain of memory, with 7 subjects (4 CTCL and 3 psoriasis) out of 39 (17.9%) demonstrating clinical impairment. Additionally, 5 subjects (4 CTCL and 1 psoriasis) out of 39 (12.8%) were impaired in the animal naming test.

### 3.3. Psychological Profile and Health-Related Quality of Life

There were no significant differences in the mean STAI *T*-scores and BDI-II raw scores of CTCL versus psoriasis subjects (Table 1), and self-reported ratings of anxiety and depression were not clinically elevated. There were no significant differences in the HR-QOL scores of CTCL versus psoriasis subjects (Tables 1 and 3).

### 3.4. Predictors of Cognitive Function, SKINDEX-29 Scores, and Psychological Function

Linear regression was used to identify potential predictors within the sample. For all regression analyses, the cognitive or SKINDEX-29 domain served as the dependent variable, and predictors (i.e., disease duration, depression, and anxiety) were entered into the model simultaneously. Estimated intellectual functioning was an additional predictor variable entered into the regression models for SKINDEX-29. See Table 4 for regression coefficients of significant omnibus tests.

#### 3.4.1. Predictors of Cognitive Function

Separate linear regressions were conducted for each cognitive domain. The full model contained disease duration, BDI-II, STAI-state, and STAI-trait scores. The full model was a significant predictor of memory (*F* (4, 31) = 2.90, p = 0.04). Examination of individual predictors revealed that shorter disease duration was associated with worse memory. The full model was not a significant predictor of attention and processing speed, executive functioning, or MMSE total score.

To determine if SKINDEX-29 scores predicted cognitive status, separate linear regressions were conducted for each cognitive domain. The full model contained each subcategory of SKINDEX-29 (emotions, symptoms, and functioning). The full model was a significant predictor of executive functioning only (*F* (3, 35) = 6.93, *p* < 0.01). Examination of individual predictors revealed that a higher score on the functioning domain was associated with worse executive functioning.

#### 3.4.2. Predictors of Animal Naming Test

Disease duration was a significant predictor of the animal naming test (*F* (4, 34) = 4.04, *p* = 0.01), with shorter disease duration being associated with worse performance on this measure. The SKINDEX-29 symptom score was also a significant predictor of the animal naming test (*F* (3, 35) = 3.94, *p* = 0.02) with higher scores on the symptom domain being associated with a better animal naming test.

#### 3.4.3. Predictors of SKINDEX-29 Scores

Separate linear regressions were conducted for each SKINDEX-29 domain. The full model contained disease duration, estimated premorbid intellectual functioning, BDI-II, STAI-state, and STAI-trait scores. The full model was a significant predictor of emotions (*F* (5, 33) = 6.20, p < 0.001), symptoms (*F* (5, 33) = 4.46, p < 0.01), and functioning (*F* (5, 33) = 6.22, p < 0.001) scores of SKINDEX-29. Examination of individual predictors revealed a statistical trend (*p* < 0.10) for higher levels of self-reported depression to be associated with higher scores in the emotion domain, as well as a trend for higher estimated intellectual functioning to be associated with lower scores in this domain. Higher estimated intellectual functioning was associated with lower scores in the symptom domain; there was also a statistical trend for higher levels of state (acute) anxiety to be associated with lower scores in this domain. Higher estimated intellectual functioning was associated with lower scores in the functioning domain; there was a statistical trend for higher self-reported levels of depression to be associated with higher scores in this domain.

#### 3.4.4. Predictors of Psychological Function

To determine if disease duration predicted psychological status, separate linear regressions were conducted for depression, state anxiety, and trait anxiety. The full model was a significant predictor of state anxiety (*F* (1, 37) = 7.50, *p* = 0.01), with shorter disease duration being associated with higher levels of state anxiety.

## 4. Discussion

In this study, cognitive impairment was found in the domain of memory in a subset of CTCL and psoriasis subjects. Both memory and acute anxiety were adversely impacted by shorter disease duration which is speculated to be from a lack of psychological adaptation to skin disease. For the SKINDEX-29 symptoms and functioning domains, a higher estimated intellectual function predicted lower scores, translated as a better subjective HR-QOL, demonstrating that patients with stronger cognitive resources appear to cope better with the disease. Among 1,580 patients with psoriasis, planning and active coping were the coping strategies that most patients used for dealing with psychological distress followed by acceptance and positive reframing [28]. The least used coping strategies were denial, behavioral disengagement, and substance abuse. One possibility is that individuals with a higher degree of baseline cognitive resources are better equipped for positive coping strategies such as planning and active coping; however, further studies are needed to explore this speculation. This current study is limited by the small sample size as well as the cross-sectional design.

The animal naming test remains an easy-to-perform screening test for clinicians that want to evaluate early MCI. Interestingly, we found for the first time that better animal naming test performances are related to worse skin severity and longer disease duration, suggesting that dermatological patients may early experience a transitory decrease in the animal naming test due to the disease that mitigates with time and a reactive increase during flares to compensate the psychological pain (adaptive mechanism).

There is controversy in relation to cognitive disorders in patients with psoriasis and only limited information on CTCL [29–34]. In one study, mild cognitive impairment (MCI) was significantly higher among 18 out of 41 patients with moderate to severe chronic plaque psoriasis compared to controls [29]. The presence of psoriasis was found to be the only significant predictor of MCI, independent of age, gender, levels of education, smoking habit, hypertension, diabetes, and hypercholesterolemia [29].

A large database study by Pezzolo and colleagues utilized a database of patients undergoing MCI testing to study psoriasis cognition and did not find higher levels of MCI as compared to a control population [30]. MRI results were included in the studies by Pezzolo et al. and by Gisondi et al. [29], which showed no volumetric, microstructural, or focal brain differences between psoriatic patients and controls. Examining patients from within a cohort already selected for suspicion of MCI may introduce a selection bias that is different from the other studies. By contrast, our study was performed among patients that had neither a previous diagnosis of MCI nor instrumental or clinical signs that prompted an MCI evaluation.

Furthermore, drug use may interfere and even trigger MCI, so we decided to exclude patients with smoking and alcohol use, in distinction from some previous studies [31, 32].

We also included only patients in therapeutic washout to minimize the impact of therapies [29, 32, 33]. The etiology of cognitive impairment in patients with chronic dermatological conditions is uncertain but may be multifactorial. Speculation includes a common genetic background linking psoriasis to Alzheimer's disease (AD), i.e., the APOE-*ε*4 allele, cardiovascular risk factors especially the metabolic syndrome, and tumor necrosis factor-*α* because of its role in neural functions as well as in inflammation. Studies on the APPPS1 AD mouse model demonstrated increased microglia production of the IL-12 and IL-23 subunit p40 which are also increased in psoriatic lesions [14]. Inhibition of the IL-12/IL-23 pathway reduced cerebral amyloidosis and reversed cognitive deficits [14]. Moreover, IL-12/23 p40 was significantly elevated in the cerebrospinal fluid of human subjects with AD compared to controls without AD [14]. Lastly, another conjecture regarding cognitive impairment and chronic skin disease in addition to a possible connection to amyloid pathogenesis [35, 36] is pathogenesis related to skin inflammation-induced acceleration of atherosclerotic microcirculatory disease in the brain.

In this study, SKINDEX-29 scores were not significantly different between CTCL and psoriasis subjects, in contrast to previous studies that found that CTCL and psoriasis had influence on the patients' emotional well-being and HR-QOL [4, 37, 38]. The HR-QOL of 22 CTCL patients was measured with a general oncology questionnaire in addition to SKINDEX-29 [4]. More advanced-stage patients reported worse HR-QOL than early-stage patients. In another study, the HR-QOL was evaluated among 95 patients with cutaneous B-cell lymphoma, mycosis fungoides, and Sezary syndrome using the SKINDEX-29 and an oncology-specific questionnaire [37]. HR-QOL was worse in Sezary syndrome patients and among those with probable anxiety or depression and with worsening disease. SKINDEX-29 scores in this current study are compared to other skin diseases (Table 3) with variable results which may reflect differences in coping mechanisms of individual patients [4, 5]. Furthermore, our preliminary study patients displayed a gender unbalance that does not allow to generalize to different populations due to the potential gender differences in psychological/emotional coping strategies, but at the same time, these data are really specific for psoriasis and CTCL patients offering several insights toward the potential animal naming test impairment in dermatological disease early stage and a reactive increase to counteract cutaneous severity.

## 5. Conclusions

Cognitive impairment may be an associated comorbidity in CTCL and psoriasis. In particular, early in the course of the disease, patients experienced significant impacts likely because they are still in the process of developing coping mechanisms. Psychological resilience associated with higher premorbid intellectual functioning appeared to serve as a buffer, possibly due to increased ability to cope, rely on, and seek out resources. Personalized care with attention to these variables may enable better outcomes for these patients. Future studies may focus on other variables potentially impacting cognitive functioning such as therapy of CTCL patients with oral bexarotene or anti-inflammatory therapies for psoriasis.

## Figures and Tables

**Figure 1:** Difference in disease duration between psoriatic and cutaneous T-cell lymphoma (CTCL) patients.

**Figure 2:** Evaluation of the three SKINDEX-29 domains (functioning, symptoms, and emotions) in patients with psoriasis and cutaneous T-cell lymphoma (CTCL).

**Table 1:** Demographic and clinical characteristics of cutaneous T-cell lymphoma (CTCL) versus psoriasis subjects.

Characteristics	CTCL (*N* = 20)	Psoriasis (*N* = 19)	*p* value^e^
Age (years), mean ± SD (range)	67 ± 9.80 (52-88)	57 ± 10.44 (42-82)	0.01
Male, sex, *n* (%)	16 (80)	14 (74)	0.72
Caucasian, *n* (%)	19 (95)	15 (79)	0.18
Years of education, mean ± SD	15 ± 3.11	14 ± 1.95	0.38
Married, *n* (%)	17 (85)	10 (53)	0.03
Currently employed, *n* (%)	8 (40)	13 (68)	0.08
Current and previous smoker, *n* (%)	9 (45)	11 (58)	0.42
Systolic blood pressure (mm Hg), mean ± SD	137 ± 18	137 ± 13	0.98
Diastolic blood pressure (mm Hg), mean ± SD	80 ± 11	89 ± 9	0.01
Body mass index (kg/m^2^), mean ± SD	30 ± 5	30 ± 8	0.83
CTCL current stage			
In remission	7		
IA^1^	10		
IB^2^	2		
IVA^3^	1		
SWAT score, mean (range)	9 (0-87)	N.A.	
PASI score, mean (range)	NA	7 (0-28)	
Skin disease duration (years), mean ± SD (range)	13 ± 12 (1-44)	24 ± 15 (2-49)	0.01
Skin disease medication history			
Skin directed therapy, *n* (%)^a^	10 (50)	6 (32)	0.24
Systemic therapy, *n* (%)^b^	10 (50)	13 (68)	0.24
Prior treatment with oral bexarotene, *n* (%)	7 (35)	0 (0)	
Prior treatment with oral acitretin, *n* (%)	0 (0)	3 (16)	
Estimated intelligence quotient, mean ± SD^c^	106.90 ± 7.75	104.42 ± 10.00	0.39
BDI-II raw score, mean ± SD^d^	8.05 ± 8.98	7.53 ± 9.95	0.86
STAI-state *T*-score, mean ± SD	52.90 ± 15.10	45.37 ± 7.80	0.06
STAI-trait *T*-score, mean ± SD	49.30 ± 11.81	46.58 ± 8.86	0.42
SKINDEX-29 emotion score, mean ± SD	25.63 ± 24.67	31.97 ± 28.00	0.46
SKINDEX-29 symptom score, mean ± SD	26.25 ± 24.12	39.10 ± 27.93	0.13
SKINDEX-29 functioning score, mean ± SD	13.64 ± 19.78	21.38 ± 27.51	0.32

Notes: ^a^skin-directed therapy for CTCL subjects included clinical trials, phototherapy, radiation, and topical bexarotene, nitrogen mustard, and steroids. Skin-directed therapy for psoriasis subjects included clinical trials, phototherapy, tar, and topical calcipotriene, steroids, and tacrolimus. ^b^Systemic therapy for CTCL subjects included brentuximab, clinical trials, combination chemotherapy, extracorporeal photopheresis, interferon, oral bexarotene, prednisone, and vorinostat. Systemic therapy for psoriasis subjects included acitretin, apremilast, clinical trials, cyclosporine, etanercept, ixekizumab, methotrexate, steroids, and ustekinumab. ^c^The North American Adult Reading Test standard scores were used to estimate intelligence quotient. Average mean intelligence quotient is 100 with standard deviation of 15. ^d^BDI cutoff scores: 0-9: within normal limits; 10-15: minimal depression; 16-19: mild to moderate depression; 20-29: moderate to severe depression; 30+: severe depression; ^e^*p* values were calculated with *t*-Student to compare means of two independent samples (CTCL and psoriasis) using a freedom degree of 38 (number of observations–groups considered). 1: less than 10% of the skin is covered in red patches or plaques, and there is no blood, lymph node, or internal organ involvement. 2: 10% or more of the skin is covered in patches or plaques, and there is no blood, lymph node, or internal organ involvement. 3: most of the skin is reddened, and cancer is found in the blood; cancer may have spread to the lymph nodes but does not involve other internal organs. Abbreviations: BDI-II: Beck Depression Inventory-II; NA: not applicable; PASI: Psoriasis Area and Severity Index; STAI: State-Trait Anxiety Inventory; SWAT: modified Severity-Weighted Assessment Tool.

**Table 2:** Neuropsychological tests focused on cognitive performance of cutaneous T-cell lymphoma (CTCL) versus psoriasis subjects.

Cognitive domain/test^a^	CTCL (*N* = 20)	Psoriasis (*N* = 19)	*p* value^b^
Memory *T*-score, mean ± SD	42.37 ± 12.01	45.06 ± 12.26	0.51
Attention/processing speed *T*-score, mean ± SD	47.14 ± 5.02	46.95 ± 4.47	0.93
Executive functioning *T*-score, mean ± SD	50.33 ± 6.24	48.48 ± 6.10	0.36
Semantic fluency *T*-score, mean ± SD	46.55 ± 11.01	51.32 ± 12.93	0.22

Notes: ^a^all scores are standardized *T*-scores based on normative data, unless otherwise noted. Age was controlled for in analysis using raw scores. ^b^*p* values were obtained with *t*-Student to compare means of two independent samples (CTCL and psoriasis) using a freedom degree of 38 (number of observations–groups considered).

**Table 3:** SKINDEX-29 domain scores of various dermatologic diseases.

Skin disease	Number of subjects	SKINDEX-29 emotions, mean score ± SD	SKINDEX-29 symptoms, mean score ± SD	SKINDEX-29 functioning, mean score ± SD	Reference
CTCL (*N* = 20)	20	25.6 ± 24.7	26.3 ± 24.1	13.6 ± 19.8	Current study
Psoriasis (*N* = 19)	19	31.9 ± 28.0	39.1 ± 27.9	21.4 ± 27.5	Current study
CTCL	22	23.9 ± 8.9	19.1 ± 7.2	24.2 ± 10.4	Demierre, et al. ^4^
Psoriasis	44	39 ± 27	42 ± 21	23 ± 27	Chren et al. ^5^
Eczematous dermatitis	102	41 ± 27	48 ± 23	26 ± 26	Chren et al. ^5^
Acne vulgaris	63	41 ± 25	30 ± 19	16 ± 16	Chren et al. ^5^
Warts	24	39 ± 27	42 ± 21	23 ± 27	Chren et al. ^5^
Other benign growths	76	21 ± 21	22 ± 20	9 ± 17	Chren et al. ^5^

Notes: higher scores in SKINDEX-29 indicate worse health-related quality of life. Legend: BDI-II: Beck Depression Inventory-II; CTCL: cutaneous T-cell lymphoma; STAI: State-Trait Anxiety Inventory.

**Table 4:** Regression coefficients for predictors of cognitive function and SKINDEX-29 domain scores in cutaneous T-cell lymphoma and psoriasis subjects.

Coefficients/predictor variables	*B*	SE	*β*	*t*-statistic	*p* value
Memory (*n* = 36)					
Skin disease duration (years)	0.41	0.14	0.49	2.93	0.01
BDI-II raw score	-0.25	0.30	-0.20	-0.84	0.41
STAI-state *T*-score	0.02	0.21	0.02	0.08	0.94
STAI-trait *T*-score	0.11	0.29	0.10	0.38	0.71
Animal naming test					
Skin disease duration (years)	0.28	0.13	0.33	2.13	0.04
BDI-II raw score	-0.11	0.28	-0.08	-0.37	0.71
STAI-state *T*-score	-0.16	0.97	-0.16	-0.80	0.43
STAI-trait *T*-score	-0.17	0.28	-0.15	-0.63	0.53
Executive function					
SKINDEX-29 emotion score	-0.21	0.07	-0.09	-0.30	0.77
SKINDEX-29 symptom score	0.06	0.05	0.25	1.13	0.27
SKINDEX-29 functioning score	-0.18	0.08	-0.71	-2.24	0.03
Animal naming test					
SKINDEX-29 emotion score	-0.23	0.15	-0.49	-1.52	0.14
SKINDEX-29 symptom score	0.28	0.11	0.61	2.49	0.02
SKINDEX-29 functioning score	-0.18	0.18	-0.35	-1.02	0.31
SKINDEX-29 emotions					
Skin disease duration (years)	-0.14	0.26	-0.07	-0.52	0.61
BDI-II raw score	1.07	0.60	0.38	1.79	0.08
STAI-state *T*-score	-0.18	0.38	-0.08	-0.46	0.65
STAI-trait *T*-score	0.43	0.53	0.17	0.80	0.43
NAART standard score	-0.86	0.46	-0.29	-1.89	0.07
SKINDEX-29 symptoms					
Skin disease duration (years)	-0.28	0.28	-0.15	-0.99	0.34
BDI-II raw score	1.04	0.65	0.37	1.60	0.12
STAI-state *T*-score	-0.78	0.41	-0.37	-1.90	0.07
STAI-trait *T*-score	0.12	0.58	0.05	0.21	0.83
NAART standard score	-1.31	0.50	-0.44	-2.62	0.01
SKINDEX-29 functioning					
Skin disease duration (years)	-0.30	0.24	-0.18	-1.28	0.21
BDI-II raw score	1.07	0.55	0.42	1.97	0.06
STAI-state *T*-score	-0.43	0.34	-0.23	-1.25	0.22
STAI-trait *T*-score	0.16	0.49	0.07	0.33	0.75
NAART standard score	-1.04	0.42	-0.39	-2.49	0.02
State anxiety					
Skin disease duration (years)	-0.36	0.13	-0.41	-2.74	0.01

Legend: BDI-II: Beck Depression Inventory-II; NAART: North American Adult Reading Test; STAI: State-Trait Anxiety Inventory.

## Data Availability

Data could be accessed in a private repository upon request to Prof. Kevin Cooper (kdc@case.edu).
